# Integrated Bioinformatics Analysis for Identifying the Significant Genes as Poor Prognostic Markers in Gastric Adenocarcinoma

**DOI:** 10.1155/2022/9080460

**Published:** 2022-06-11

**Authors:** Yamei Li, Yan Luo, Qiang Tian, Yu Lai, Lei Xu, Hailong Yun, Yang Liang, Dandan Liao, Rui Gu, Liye Liu, Mu Yuan, Yijiao Li, Yufan Li, Mingze Lu, Xin Yong, Hua Zhang

**Affiliations:** ^1^Department of Laboratory Medicine, West China Hospital of Sichuan University, Chengdu 610041, China; ^2^Department of Pathology, General Hospital of Western Theater Command, Chengdu 610083, China; ^3^Department of Oncology, The Fifth People's Hospital of Nanchong (People's Hospital of Gaoping District Nanchong), Nanchong 637000, China; ^4^Laboratory of Basic Medicine, General Hospital of Western Theater Command, Chengdu 610083, China; ^5^Department of General Surgery, General Hospital of Western Theater Command, Chengdu 610083, China; ^6^Department of Scientific Research & Training, General Hospital of Western Theater Command, Chengdu 610083, China; ^7^Department of Anesthesiology, The People's Hospital of Leshan, Leshan 614000, China; ^8^Department of Human Resources, General Hospital of Western Theater Command, Chengdu 610083, China; ^9^Department of Gastroenterology, General Hospital of Western Theater Command, Chengdu 610083, China; ^10^State Key Laboratory of Biotherapy, Sichuan University, Chengdu 610041, China

## Abstract

Gastric adenocarcinoma (GAC) is the most common histological type of gastric cancer and imposes a considerable health burden globally. The purpose of this study was to identify significant genes and key pathways participated in the initiation and progression of GAC. Four datasets (GSE13911, GSE19826, GSE54129, and GSE79973) including 171 GAC and 77 normal tissues from Gene Expression Omnibus (GEO) database were collected and analyzed. Through integrated bioinformatics analysis, we obtained 69 commonly differentially expressed genes (DEGs) among the four datasets, including 20 upregulated and 49 downregulated genes. The prime module in protein-protein interaction network of DEGs, including ADAMTS2, COL10A1, COL1A1, COL1A2, COL8A1, BGN, and SPP1, was enriched in protein digestion and absorption, ECM-receptor interaction, focal adhesion, PI3K-Akt signaling pathway, and amoebiasis. Furthermore, expression and survival analysis found that all seven hub genes were highly expressed in GAC tissues and 6 of them (except for SPP1) were able to predict poor prognosis of GAC. Finally, we verified the 6 high-expressed hub genes in GAC tissues via immunohistochemistry, Western blot, and RNA quantification analysis. Altogether, we identified six significantly upregulated DEGs as poor prognostic markers in GAC based on integrated bioinformatical methods, which could be potential molecular markers and therapeutic targets for GAC patients.

## 1. Introduction

Gastric adenocarcinoma (GAC), the predominant histological type of gastric cancer, is the fifth most common cancer ranked after lung, breast, colorectal, and prostate cancers [1, 2]. GAC, also known as stomach adenocarcinoma (STAD), has increased more than 1,000,000 new cases and led to deaths of more than 768,000 people worldwide in 2020 [3]. Although improvements in endoscopic, surgical, and systemic treatments have been made for decades, the mortality rate of GAC is still high and the global 5-year survival rates remain unsatisfactory [1, 4]. Thus, GAC still imposes a considerable health burden globally.

Although the global 5-year survival rates are relatively low, the rates in Japan and South Korea are far more optimistic [5, 6], owing to early detection and screening efforts in these Asian countries [7]. Furthermore, it is reported that the 5-year survival rate of early-stage T1 GAC (according to the TNM classification of malignant tumors) is ∼95%, while advanced-stage GAC (which cannot be surgically treated) has a median survival of ∼9-10 months [8, 9], which further emphasizes the critical importance of early detection and diagnosis.

Molecular markers are vital for early detection of cancer [10–12]. To date, several biomarkers have been used for the diagnosis and determination of the clinical stage of GAC. Among them, carcinoembryonic antigen (CEA), carbohydrate antigen 19-9 (CA19-9), and erb-b2 receptor tyrosine kinase 2 (HER2) are the most frequently used biomarkers for GAC in clinical setting [13, 14]. However, due to the insufficient specificity and sensitivity of the current markers, novel specific and sensitive molecular markers are still on urgent demand, especially in the field of early diagnosis and prognosis [13–15]. Bioinformatics analysis is a powerful and comprehensive tool for analyzing gene expression data from multiple datasets, which is perfect for excavating the potential molecular markers laid in Gene Expression Omnibus (GEO) and The Cancer Genome Atlas (TCGA) datasets. Therefore, in the current study, we mainly focused on exploring the commonly differential expressed genes among different GEO datasets. Gene ontology (GO) and KEGG enrichment analysis were further conducted to identify the hub genes and key pathways enriched in the commonly DEGs. Protein-protein interaction (PPI) network of the DEGs was constructed, and core genes were determined via the Cytoscape Molecular Complex Detection (MCODE). In addition, DAVID, GEPIA, and Kaplan–Meier plotter were applied to re-analyze the expression and survival information of the core genes, respectively [16, 17]. Finally, immunohistochemistry, Western blot, and RNA quantification analysis were performed to validate the expressions of the identified genes in GAC tissue samples.

## 2. Materials and Methods

### 2.1. Microarray Data Information

NCBI-GEO is a free public database and provides us with gene expression profile of numerous cancers. The following criteria were used to screen the datasets and ensure relevant data were recorded: (I) the sample includes gastric adenocarcinoma and normal tissues; (II) the study type is expression profiling by array; (III) the species is limited to Homo sapiens; (IV) access to raw data is allowed. We obtained the gene expression profiles of GSE13911, GSE19826, GSE54129, and GSE79973 in gastric adenocarcinoma and paired normal tissues. Microarray data of GSE13911, GSE19826, GSE54129, and GSE79973 were all on account of GPL570 platforms ([HG-U133_Plus_2] Affymetrix Human Genome U133 Plus 2.0 Array) which included a total of 171 GAC tissues and 77 normal tissues.

### 2.2. DEGs Identification

Background correction and normalization were conducted through robust multi-array average (RMA) and Microarray Suite (MAS) approach. The GEO2R online tools [18] were used to identify DEGs between the GAC specimen and normal specimen with |log_2_FC| > 2 and an adjusted *P* value <0.05 [16–18]. Then, the raw data were analyzed in Venn software online to identify the commonly DEGs among the original four datasets. The DEGs with log_2_FC > 0 were considered as upregulated genes, while the DEGs with log_2_FC ＜ 0 were considered as downregulated genes [16, 17].

### 2.3. GO and Pathway Enrichment Analysis

The functions and pathways enrichment of candidate DEGs were analyzed using DAVID (the Database for Annotation, Visualization and Integrated Discovery, https://david.ncifcrf.gov/) [19], which is an online bioinformatic tool with the function of integrating the GO and pathway enrichment analysis [20, 21]. Through DAVID, we identified the unique biological properties of the commonly DEGs and visualized the DEGs enrichment of molecular function (MF), cellular component (CC), biological process (BP), and Kyoto Encyclopedia of Gene and Genome (KEGG) pathways (*P* < 0.05) [16, 17].

### 2.4. Integration of PPI Network and Modular Analysis

STRING (Search Tool for the Retrieval of Interacting Genes, https://cn.string-db.org/) online tool [22] was used to evaluate the PPI information of DEGs. Then, the STRING app in Cytoscape [23] was employed to examine the potential correlation between these DEGs (maximum number of interactors = 0 and confidence score ≥0.4). In addition, the MCODE app in Cytoscape was used to identify the modules and hub genes of the PPI network (degree cutoff = 2, max. depth = 100, *k-*core = 2, and node score cutoff = 0.2) [16, 17]. PPI network properties, such as node degree and betweenness centrality, were visualized by shape size and label font size, respectively.

### 2.5. Survival and RNA Sequencing Expression Analysis

Kaplan–Meier plotter is a common website tool (https://kmplot.com/), which contains considerable information among several cancers, including breast and gastric cancer [24]. The survival analysis was conducted by Kaplan–Meier plotter, and the log rank *P* value and hazard ratio (HR) with 95% confidence intervals were computed and shown on the plot. To validate these DEGs with significant expression pattern, we applied the GEPIA (Gene Expression Profiling Interactive Analysis, https://gepia.cancer-pku.cn/) website to analyze the data of RNA sequencing expression based on the GTEx projects and TCGA datasets [25].

### 2.6. Immunohistochemical (IHC) Staining

IHC staining was performed to detect the protein level of certain genes in GAC and normal human tissue samples and performed according to the standard protocols using following antibodies: anti-ADAMTS2 (bs-5858R, 1 : 500), anti-COL10A1 (BA2023, 1 : 400), anti-COL1A1 (BA0325, 1 : 400), anti-COL1A2 (BM4017, 1 : 100), anti-COL8A1 (bs-7529R, 1 : 500), and anti-BGN (bs-7552R, 1 : 500).

### 2.7. Western Blot

GAC and adjacent normal tissue samples were grinded and lysed with RIPA buffer supplemented with protease inhibitor cocktail. Protein concentrations of the extracts were measured with BCA assay. The Western blot analysis was performed according to the standard protocols using the above antibodies.

### 2.8. RNA Quantification

Total RNA was extracted from GAC and adjacent normal tissues with TRIzol reagent (Invitrogen) and reverse-transcribed using PrimeScript™ RT reagent kit (Takara). Quantitative real-time PCR analysis was performed on LightCycler (Roche) with TB Green® Premix Ex Taq™ II (Takara). Data were normalized to *GAPDH* expression. The primers used for real-time PCR were as follows: *GAPDH* (forward: 5′-GGA GCG AGA TCC CTC CAA AAT-3′, reverse: 5′-GGC TGT TGT CAT ACT TCT CAT GG-3′), *ADAMTS2* (forward: 5′-GTG CAT GTG GTG TAT CGC C-3′, reverse: 5′-AGG ACC TCG ATG TTG TAG TCA-3′), *COL10A1* (forward: 5′-CAT AAA AGG CCC ACT ACC CAA C-3′, reverse: 5′-ACC TTG CTC TCC TCT TAC TGC-3′), *COL1A1* (forward: 5′-GAG GGC CAA GAC GAA GAC ATC-3′, reverse: 5′-CAG ATC ACG TCA TCG CAC AAC-3′), *COL1A2* (forward: 5′-GGC CCT CAA GGT TTC CAA GG-3′, reverse: 5′-CAC CCT GTG GTC CAA CAA CTC-3′), *COL8A1* (forward: 5′-GCT GCC ACC TCA AAT TCC TC-3′, reverse: 5′-CTT TCT TGG GTA CGG CTT CCT-3′), and *BGN* (forward: 5′-GAG ACC CTG AAT GAA CTC CAC C-3′, reverse: 5′-CTC CCG TTC TCG ATC ATC CTG-3′).

## 3. Results

### 3.1. Identification of DEGs in Gastric Adenocarcinoma

GEO2R online tool was used to determine the DEGs from GSE13911, GSE19826, GSE54129, and GSE79973, which resulted in 484, 388, 971, and 524 DEGs, respectively (Figure 1(a)) (|log_2_FC| ＞ 2 and adjust *P* value ＜0.05). Then, the commonly DEGs among the above four datasets were identified by Venn diagram software. Results showed that a total of 69 commonly DEGs were identified, including 20 upregulated genes (log_2_FC ＞ 2) and 49 downregulated genes (log_2_FC ＜ −2) in GAC tissues (Figures 1(b) and 1(c) and Table 1).

### 3.2. GO and KEGG Analysis of DEGs in Gastric Adenocarcinoma

In order to examine the biological properties of the 69 DEGs, DAVID software was applied to conduct GO and KEGG analysis. Results of GO analysis indicated that (1) for biological processes (BP), upregulated DEGs were particularly enriched in endodermal cell differentiation, collagen fibril organization, protein heterotrimerization, skin morphogenesis, and cell adhesion, and downregulated DEGs in digestion, potassium ion import, oxidation-reduction process, and bicarbonate transport (Figure 2(a)); (2) for cell component (CC), upregulated DEGs were significantly enriched in extracellular space, collagen trimer, collagen type I trimer, and proteinaceous extracellular matrix, and downregulated DEGs in extracellular space, lysosome, apical plasma membrane, integral component of plasma membrane, and integral component of membrane (Figure 2(b)); (3) for molecular function (MF), upregulated DEGs were enriched in extracellular matrix structural constituent and heparin binding, and downregulated DEGs in inward rectifier potassium channel activity, hydrogen:potassium-exchanging ATPase activity, and G-protein activated inward rectifier potassium channel activity (Figure 2(c) and Table 2, *P* < 0.05).

Results of KEGG analysis showed that upregulated DEGs were particularly enriched in ECM-receptor interaction, focal adhesion, protein digestion and absorption, PI3K-Akt signaling pathway, amoebiasis, and platelet activation (Figure 3(a)), while downregulated DEGs in gastric acid secretion, retinol metabolism, chemical carcinogenesis, collecting duct acid secretion, glycolysis/gluconeogenesis, drug metabolism-cytochrome P450, metabolism of xenobiotics by cytochrome P450, and metabolic pathways (Figure 3(b) and Table 3, *P* < 0.05).

### 3.3. PPI Network and Modular Analysis of DEGs

The DEGs PPI network complex was constructed via Cytoscape software. Results showed that 44 DEGs including 16 upregulated and 28 downregulated genes were enrolled, and 75 edges were formed (Figure 4(a)). There were 25 DEGs which were not included into the DEGs PPI network. Then, we applied Cytoscape MCODE to further analyze the prime module and ADAMTS2, COL10A1, COL1A1, COL1A2, COL8A1, BGN, and SPP1 were identified among the 44 nodes. Results also showed that the above seven hub nodes were all upregulated genes (Figure 4(b)).

### 3.4. Re-Analysis of Seven Hub Genes by KEGG Pathway Enrichment

To further understand the possible enriched pathways of the seven hub DEGs, KEGG pathway enrichment was re-analyzed via DAVID. Results showed that seven core genes were significantly enriched in several cancer-related pathways. In detail, COL1A2, COL1A1, and COL10A1 were enriched in protein digestion and absorption; COL1A2, COL1A1, and SPP1 were enriched in ECM-receptor interaction, focal adhesion, and PI3K-Akt signaling pathway; COL1A2 and COL1A1 were further enriched in amoebiasis (Figure 5 and Table 4, *P* < 0.05).

### 3.5. Analysis of Hub Genes via the GEPIA and Kaplan–Meier Plotter

To further validate the significance of the seven central genes, GEPIA and Kaplan–Meier plotter online tools were utilized to identify the expression data and survival data, respectively. GEPIA expression data showed that all seven hub genes were highly expressed in GAC tissues compared to normal tissues (Figure 6 and Table 5, *P* < 0.05). Kaplan–Meier plotter survival data showed that high expression of ADAMTS2, COL10A1, COL1A1, COL1A2, COL8A1, and BGN had a significantly worse survival probability, while high expression of SPP1 showed no effect on patient survival (Figure 7 and Table 6, *P* < 0.05).

### 3.6. Validation of the Expression Levels of Six Core Genes in GAC Patients

Finally, we detected the expression levels of the above six genes in GAC specimens and adjacent normal specimens by immunohistochemistry (Figure 8(a)), Western blot (Figure 8(b)), and RNA quantification (Figure 8(c)) analysis. Results showed that ADAMTS2, COL10A1, COL1A1, COL1A2, COL8A1, and BGN were highly expressed in GAC tissues compared to adjacent normal tissues (Figure 8), consistent with the GEPIA expression data.

## 4. Discussion

Gastric adenocarcinoma is a lethal malignance cancer. In this study, we applied bioinformatical methods on the basis of four gene expression profile datasets to identify more useful prognostic molecular markers in GAC. A total of 171 GAC specimens and 77 normal specimens were enrolled. First, we revealed a total of 69 commonly DEGs via GEO2R and Venn software (|log_2_FC| ＞ 2 and adjust *P* value ＜0.05), including 20 upregulated and 49 downregulated DEGs. Second, GO and KEGG pathway enrichment analysis showed that 20 upregulated genes enriched in endodermal cell differentiation, protein heterotrimerization, ECM-receptor interaction, focal adhesion, protein digestion and absorption, PI3K-Akt signaling pathway, amoebiasis, and platelet activation, while 49 downregulated genes enriched in digestion, potassium ion import, oxidation-reduction process, bicarbonate transport, inward rectifier potassium channel activity, hydrogen:potassium-exchanging ATPase activity, gastric acid secretion, retinol metabolism, and metabolic pathways (*P* < 0.05). Third, DEGs PPI network complex of 44 nodes and 75 edges was constructed via Cytoscape software and prime module analysis identified 7 hub genes (ADAMTS2, COL10A1, COL1A1, COL1A2, COL8A1, BGN, and SPP1), which were all upregulated genes and were significantly enriched in several cancer-related pathways. Furthermore, GEPIA analysis showed that all the seven hub genes were highly expressed in GAC tissues (*P* < 0.05). In addition, Kaplan–Meier plotter analysis showed that high expression of ADAMTS2, COL10A1, COL1A1, COL1A2, COL8A1, and BGN had a significantly worse survival probability (*P* < 0.05), while SPP1 had no significance (*P* > 0.05). Finally, the 6 highly expressed core genes were validated via immunohistochemistry, Western blot, and RNA quantification analysis in tissue samples. Altogether, we identified six significant upregulated genes as poor prognosis markers in gastric adenocarcinoma via bioinformatical analysis, which could be potential new molecular markers and effective targets for early detection and further research.

The hub genes in the main module of the PPI network of the commonly DEGs are mainly associated with protein digestion and absorption, ECM-receptor interaction, focal adhesion, PI3K-Akt signaling pathway, and amoebiasis. The family of collagen genes (CLO10A1, COL1A1, COL1A2, etc.) is tightly clustered and participates in the above cancer-related pathways. Furthermore, studies have demonstrated the close relation between collagen genes and gastric adenocarcinoma, including COL10A1, COL1A1, COL1A2, and COL8A1. What's more, it is well known that PI3K-Akt signaling pathway (COL1A2, COL1A1, etc.) plays a vital role in the cell cycle and is activated in various cancers, including GAC [26]. For ADAMTS2, a member of the ADAMTS family is a procollagen N-proteinase [27]. Researches have shown that ADAMTS2 participated in major biological pathways and human disorders [28], but the relation between ADAMTS2 and GAC has rarely been studied [27]. Furthermore, BGN, a key member of the small leucine-rich proteoglycan family, has been shown to participate in many cancers and is associated with poor prognosis in cancer patients, including gastric adenocarcinoma [29]. The results and related studies have provided solid evidence to prove the relation between the hub genes along with the enriched pathways and GAC.

Expression and survival analysis have demonstrated that ADAMTS2, COL10A1, COL1A1, COL1A2, COL8A1, and BGN are all highly expressed in GAC and their high expression has a significantly worse survival. Previous studies have also showed that the abnormal expression level of the six hub genes could be indicators of the initiation, progression, and clinical outcome of GAC. Till now, little is known about the exact mechanism of the six genes in GAC initiation and progression. In our study, we have provided more helpful information and direction for the future study of GAC via integrated bioinformatical methods, which would be new perspective and clues for early detection and diagnosis of GAC.

## 5. Conclusion

Altogether, our bioinformatics analysis study identified six upregulated DEGs (ADAMTS2, COL10A1, COL1A1, COL1A2, COL8A1, and BGN) between gastric adenocarcinoma and normal tissues based on four different microarray datasets. Results showed that these six genes were poor prognostic markers, which may play key roles in the initiation and progression of GAC. These data presented in this study may provide new perspectives and clues into the early detection and therapeutic targets of GAC. However, more experiments and details are needed to verify the prediction and underlying mechanisms in the near future.

## Figures and Tables

**Figure 1:** Identification of 69 commonly differentially expressed genes (DEGs) among the four datasets (GSE13911, GSE19826, GSE54129, and GSE79973) through Venn diagram software (available online: https://bioinformatics.psb.ugent.be/webtools/Venn/). (a) Volcano plot of DEGs from the four datasets. (b) Twenty DEGs were upregulated among the four datasets (log_2_FC ＞ 0). (c) Forty-nine DEGs were downregulated among the four datasets (log_2_FC ＜ 0). Different colors represented different datasets in B and C.

**Figure 2:** Gene ontology analysis of commonly DEGs in gastric adenocarcinoma. DAVID software was applied to conduct gene ontology. Biological processes (BP) (a), cell component (CC) (b), and molecular function (MF) (c) of the up/downregulated DEGs were shown (*P* < 0.05).

**Figure 3:** KEGG analysis of commonly DEGs in gastric adenocarcinoma. KEGG analysis of upregulated DEGs (a) and downregulated DEGs (b) was shown (*P* < 0.05).

**Figure 4:** DEGs PPI network was constructed by Cytoscape software. (a) There were a total of 44 nodes and 75 edges in the DEGs PPI network complex. The nodes meant proteins; the edges meant the interaction between proteins; red circles meant upregulated DEGs; and green circles meant downregulated DEGs. (b) Modular analysis via Cytoscape software (degree cutoff = 2, max. depth = 100, *k*-core = 2, and node score cutoff = 0.2). Seven central nodes were screened. Circle size represents node degree, and label font size represents betweenness centrality.

**Figure 5:** KEGG re-analysis of the seven hub genes.

**Figure 6:** Expression level of the seven hub genes in gastric adenocarcinoma patients compared to healthy people. To further validate the expression level between GAC patients and normal people, seven genes were analyzed via GEPIA website. All seven genes were significantly highly expressed in GAC specimen compared to normal specimen (^*∗*^*P* < 0.05). Red color meant GAC tissues (*n* = 408), and grey color meant normal tissues (*n* = 211).

**Figure 7:** Prognostic information of the seven hub genes. Kaplan–Meier plotter online tools were used to analyze the prognostic information of the seven hub genes. High expression of ADAMTS2, COL10A1, COL1A1, COL1A2, COL8A1, and BGN had a significantly worse survival rate (*P* < 0.05).

**Figure 8:** Validation of expression levels of ADAMTS2, COL10A1, COL1A1, COL1A2, COL8A1, and BGN in GAC patients. To further validate the expression level in GAC patients, six genes were re-analyzed via immunohistochemistry (a), Western blot (b), and real-time PCR (c) analysis. Representative images of IHC staining were shown. Scale bar, 200 *μ*m. Real-time PCR data were normalized to *GAPDH* expression. All six genes were highly expressed in GAC tissue compared to adjacent normal tissue.

**Table 1:** All 69 commonly differentially expressed genes (DEGs) were identified from four profile datasets, including 20 upregulated genes and 49 downregulated genes in the gastric adenocarcinoma tissues compared to normal tissues.

DEGs	Genes name
Upregulated	IGF2BP3 SULF1 FAP RARRES1 INHBA SPP1 COL1A1 COL10A1 FNDC1 COL11A1 CEMIP CTHRC1 THBS2 BGN COL1A2 CST1 MFAP2 ADAMTS2 WISP1 COL8A1

Downregulated	CNTN3 LIPF TRIM74///TRIM73 CAPN13 FBP2 AKR1B10 B4GALNT3 CYP2C18 ALDH3A1 ATP4A UGT2B15 KIAA1324 GKN1 ADGRG2 RDH12 GIF CA2 GATA5 ATP4B MAL CAPN9 SLC26A9 ESRRG ADTRP VSTM2A SSTR1 ACER2 MFSD4A DPCR1 ADH7 VSIG1 PGC KCNE2 SOSTDC1 TPCN2 CA9 MUC5AC VSIG2 SPINK7 TMED6 SCNN1B LINC00982 HPGD PSAPL1 CWH43 KCNJ16 KCNJ15 GKN2 CXCL17

**Table 2:** Gene ontology analysis of differentially expressed genes in gastric adenocarcinoma.

Expression	Category	Term	Count	%	*P*-value	FDR
Upregulated	GOTERM_BP_DIRECT	GO:0035987∼endodermal cell differentiation	3	15.0	2.41*E* − 04	0.277424
	GOTERM_BP_DIRECT	GO:0030199∼collagen fibril organization	3	15.0	3.59*E* − 04	0.413041
	GOTERM_BP_DIRECT	GO:0070208∼protein heterotrimerization	2	10.0	0.007132	7.921921
	GOTERM_BP_DIRECT	GO:0043589∼skin morphogenesis	2	10.0	0.007132	7.921921
	GOTERM_BP_DIRECT	GO:0007155∼cell adhesion	3	15.0	0.008542	9.418433
	GOTERM_CC_DIRECT	GO:0005615∼extracellular space	8	40.0	4.61*E* − 05	0.038561
	GOTERM_CC_DIRECT	GO:0005581∼collagen trimer	3	15.0	0.001285	1.069804
	GOTERM_CC_DIRECT	GO:0005584∼collagen type I trimer	2	10.0	0.002491	2.064654
	GOTERM_CC_DIRECT	GO:0005578∼proteinaceous extracellular matrix	3	15.0	0.014327	11.37209
	GOTERM_MF_DIRECT	GO:0005201∼extracellular matrix structural constituent	3	15.0	5.25*E* − 04	0.415248
	GOTERM_MF_DIRECT	GO:0008201∼heparin binding	2	10.0	0.087398	51.56318

Downregulated	GOTERM_BP_DIRECT	GO:0007586∼digestion	5	10.2	1.81*E* − 05	0.023045
	GOTERM_BP_DIRECT	GO:0010107∼potassium ion import	4	8.2	4.56*E* − 05	0.058116
	GOTERM_BP_DIRECT	GO:0055114∼oxidation-reduction process	7	14.3	0.003333	4.16404
	GOTERM_BP_DIRECT	GO:0015701∼bicarbonate transport	3	6.1	0.005406	6.671731
	GOTERM_CC_DIRECT	GO:0005615∼extracellular space	11	22.4	0.001646	1.61346
	GOTERM_CC_DIRECT	GO:0005764∼lysosome	5	10.2	0.002499	2.44067
	GOTERM_CC_DIRECT	GO:0016324∼apical plasma membrane	5	10.2	0.006137	5.897225
	GOTERM_CC_DIRECT	GO:0005887∼integral component of plasma membrane	10	20.4	0.008007	7.631398
	GOTERM_CC_DIRECT	GO:0016021∼integral component of membrane	22	44.9	0.009103	8.634041
	GOTERM_MF_DIRECT	GO:0005242∼inward rectifier potassium channel activity	3	6.1	7.31*E* − 04	0.820368
	GOTERM_MF_DIRECT	GO:0008900∼hydrogen:potassium-exchanging ATPase activity	2	4.1	0.00603	6.584128
	GOTERM_MF_DIRECT	GO:0015467∼G-protein activated inward rectifier potassium channel activity	2	4.1	0.019965	20.31405

**Table 3:** KEGG pathway analysis of differentially expressed genes in gastric adenocarcinoma.

Expression	Term	Count	%	*P*-value	Genes
Upregulated	ptr04512:ECM-receptor interaction	5	25.0	8.56*E* − 07	COL1A2, COL1A1, THBS2, COL11A1, SPP1
	ptr04510:focal adhesion	5	25.0	2.60*E* − 05	COL1A2, COL1A1, THBS2, COL11A1, SPP1
	ptr04974:protein digestion and absorption	4	20.0	5.98*E* − 05	COL1A2, COL1A1, COL11A1, COL10A1
	ptr04151:PI3K-Akt signaling pathway	5	25.0	1.78*E* − 04	COL1A2, COL1A1, THBS2, COL11A1, SPP1
	ptr05146:amoebiasis	3	15.0	0.004694	COL1A2, COL1A1, COL11A1
	ptr04611:platelet activation	3	15.0	0.00728	COL1A2, COL1A1, COL11A1

Downregulated	hsa04971:gastric acid secretion	6	12.2	2.68*E* − 06	KCNJ16, KCNJ15, ATP4A, ATP4B, KCNE2, CA2
	hsa00830:retinol metabolism	4	8.2	0.001043	RDH12, CYP2C18, ADH7, UGT2B15
	hsa05204:chemical carcinogenesis	4	8.2	0.001989	CYP2C18, ADH7, UGT2B15, ALDH3A1
	hsa04966:collecting duct acid secretion	3	6.1	0.003265	ATP4A, ATP4B, CA2
	hsa00010:glycolysis/gluconeogenesis	3	6.1	0.019041	ADH7, FBP2, ALDH3A1
	hsa00982:drug metabolism—cytochrome P450	3	6.1	0.019581	ADH7, UGT2B15, ALDH3A1
	hsa00980:metabolism of xenobiotics by cytochrome P450	3	6.1	0.022951	ADH7, UGT2B15, ALDH3A1
	hsa01100:metabolic pathways	9	18.4	0.029288	RDH12, CYP2C18, ACER2, AKR1B10, ADH7, FBP2, UGT2B15, ALDH3A1, LIPF

**Table 4:** Re-analysis of seven selected genes via KEGG pathway enrichment.

Pathway ID	Name	Count	%	*P*-value	Genes
cfa04974	Protein digestion and absorption	3	42.9	4.55*E* − 04	COL1A2, COL1A1, COL10A1
cfa04512	ECM-receptor interaction	3	42.9	4.89*E* − 04	COL1A2, COL1A1, SPP1
cfa04510	Focal adhesion	3	42.9	0.002751	COL1A2, COL1A1, SPP1
cfa04151	PI3K-Akt signaling pathway	3	42.9	0.00721	COL1A2, COL1A1, SPP1
cfa05146	Amoebiasis	2	28.6	0.046382	COL1A2, COL1A1

**Table 5:** Validation of seven hub genes via GEPIA.

Category	Genes
Genes with high expression in GAC (*P* < 0.05)	ADAMTS2 COL10A1 COL1A1 COL1A2 COL8A1 BGN SPP1

**Table 6:** The prognostic information of the seven key candidate genes.

Category	Genes
Genes with significantly worse survival (*P* < 0.05)	ADAMTS2 COL10A1 COL1A1 COL1A2 COL8A1 BGN
Genes without significantly survival (*P* > 0.05)	SPP1

## Data Availability

The dataset supporting our findings is available at the following website: https://www.ncbi.nlm.nih.gov/geo/. All data generated or analyzed during this study are available from the corresponding author upon reasonable request.

## Abbreviations

GAC: Gastric adenocarcinoma
GEO: Gene Expression Omnibus
DEGs: Differentially expressed genes
PPI: Protein-protein interaction
DAVID: The Database for Annotation, Visualization and Integrated Discovery
GO: Gene ontology
KEGG pathways: Kyoto Encyclopedia of Gene and Genome pathways
STRING: Search Tool for the Retrieval of Interacting Genes
MCODE: Molecular Complex Detection
GEPIA: Gene Expression Profiling Interactive Analysis
TCGA: The Cancer Genome Atlas
ADAMTS2: ADAM metallopeptidase with thrombospondin type 1 motif 2
COL10A1: Collagen type X alpha 1 chain
COL1A1: Collagen type I alpha 1 chain
COL1A2: Collagen type I alpha 2 chain
COL8A1: Collagen type VIII alpha 1 chain
BGN: Biglycan
SPP1: Secreted phosphoprotein 1.
